# Oxyberberine Prevented Lipopolysaccharide-Induced Acute Lung Injury through Inhibition of Mitophagy

**DOI:** 10.1155/2021/6675264

**Published:** 2021-02-26

**Authors:** Runmin Zhao, Bingxia Wang, Dasheng Wang, Benhe Wu, Peiyu Ji, Dingyu Tan

**Affiliations:** Department of Emergency Medicine, Northern Jiangsu People's Hospital, Yangzhou University College of Clinical Medicine, Yangzhou 225001, China

## Abstract

Acute lung injury (ALI) is a serious respiratory syndrome characterized with uncontrolled inflammatory response. Oxyberberine has strong potential for clinical usage since it showed strong anti-inflammatory, antifungal, and antiarrhythmic effects in various diseases. In the present study, we evaluated whether oxyberberine can inhibit lipopolysaccharide- (LPS-) induced ALI *in vivo* and further evaluated the possible involvement of mitophagy *in vitro* by using A549 cells, a human lung epithelial cell line. Our *in vivo* study shows that oxyberberine significantly inhibited LPS-induced lung pathological injury and lung edema, as indicated by the changes in lung wet/dry ratio and total protein levels in the BALF in mice. Moreover, oxyberberine inhibited inflammation, as indicated by the changes of neutrophil accumulation and production of proinflammatory cytokines including tumor necrosis factor *α* (TNF-*α*), interleukin 1*β* (IL-1*β*), and IL-6 in both the lung and bronchoalveolar lavage fluid (BALF) in ALI mice. Our in vitro study shows that LPS significantly decreased the protein level of mitochondrial proteins, including cytochrome c oxidase subunit IV (COX IV), p62, and mitofusin-2 (Mfn2) in A549 cells. In addition, LPS induced significant Parkin1 translocation from cytoplasm to mitochondria. These changes were significantly inhibited by oxyberberine. Notably, the inhibitory effect of oxyberberine was almost totally lost in the presence of lysosome fusion inhibitor bafilomycin A1 (Baf), a mitophagy inhibitor. In conclusion, the present study demonstrated that oxyberberine alleviated LPS-induced inflammation in ALI via inhibition of Parkin-mediated mitophagy.

## 1. Introduction

Acute lung injury (ALI) is a disease characterized by the rapid onset of inflammatory responses, including bilateral pulmonary neutrophil infiltration, haemorrhage, hyaline membrane formation, lung edema, and hypothermia [1–3]. It is generally accepted that neutrophils that infiltrated into inflamed lungs are closely associated with the ALI occurrence. In addition, rapid alveolar injury characterized by alveolar epithelium and capillary endothelium caused airspace edema and inflammation due to increased alveolar barrier permeability which also serve as the important factors in the development of ALI [4, 5]. In humans, ALI and acute respiratory distress syndrome (a more severe form of ALI) score highly in terms of morbidity and mortality rates worldwide [6, 7]. ALI can lead to the development of pneumonia as well as sepsis. As yet, many researches have focused on finding the therapeutic strategies for ALI but the morbidity and mortality remain high. Thus, it is urgent to develop new and effective treatment for ALI to limit excessive inflammation.

Berberine is a quaternary isoquinoline alkaloid isolated from several traditional Chinese medicinal herbs such as *Coptidis chinensis* Franch. It has been wildly used as a nonprescription drug to treat gastroenteritis, colitis, diarrhea, and dysentery [8], due to its broad array of bioactivities (e.g., anti-inflammation, antidiarrheal, and anticolitis), low toxicity, and low cost [9]. *In vivo*, berberine could be metabolized into dihydroberberine, berberubine, demethyleneberberine, and jatrorrhizine by reduction, methylation, demethylation, and dehydroxylation, which exhibit similar pharmacological properties (e.g., anti-inflammatory, antioxidant, and anticolitis effects) to BBR. However, the activities of these metabolites are inferior to those of BBR. Recent studies show that berberine could be oxidized into 8-oxyberberine, namely, oxyberberine [10–12]. Of note, it was found that oxyberberine exhibits superior anti-inflammatory, antifungal, and antiarrhythmic activities to berberine [12–14]. Furthermore, another study shows that oxyberberine exhibits a superior safety profile as compared to berberine [12].

The specific removal of damaged mitochondria is defined as mitophagy. It is a process in which mitochondria is hydrolytically degraded by the lysosome, which is an essential method for maintaining cellular homeostasis and mitochondria function [15]. Among various signaling pathways involved in mitophagy, the PTEN-induced kinase 1- (PINK1-) Parkin signaling pathway is the typical mitophagy [16]. When there is a decrease in mitochondrial membrane potential, Parkin is recruited to the mitochondria and phosphorylated by PINK1 in the outer mitochondrial membrane [17]. Then, Parkin amplifies the mitophagy signal generated by PINK1, ubiquitinating mitochondrial proteins and inducing autophagic degradation of dysfunctional mitochondria [16, 18].

Lipopolysaccharide (LPS) is a glucosamine-based saccharolipid and the main element of the outer lipid membrane in *γ*-negative bacteria [19], and it has been extensively used to induce ALI animal models [6]. In the present study, we evaluated whether oxyberberine could inhibit LPS-induced ALI and the possible involvement of mitophagy.

## 2. Materials and Methods

### 2.1. Cell Culture

A549 cells, a human lung epithelial cell line, were purchased from the ATCC (Manassas, VA, USA). Cells were maintained in Dulbecco's modified Eagle medium/F12 (DMEM/F12) (Gibco, Thermo Fisher, Waltham, MA, USA), supplemented with 10% fetal bovine serum (FBS) (Gibco), 100 U/mL penicillin, and 100 *μ*g/mL streptomycin at 37°C under 5% CO_2_. LPS at 10 *μ*g/mL was used to treat A549 cells as previously described [20]. Cells were treated with lysosome function inhibitor Bafilomycin A1 (Baf) at 5 nmol/L for 30 min before stimulation with LPS [21].

### 2.2. Mice

All animal experiments were conducted in accordance with the Ethics Committee of Subei People's Hospital of Jiangsu Province. Eight- to ten-week-old male BALB/c mice were obtained from SLAC (Shanghai, China). Mice were housed under a 12 : 12 h light-dark cycle with free access to diet. Mice were randomly divided into 5 groups as follows: control, LPS, and oxyberberine (10, 20, and 50 mg/kg body weight) + LPS. Oxyberberine (Medkoo Biosciences Inc., Morrisville, NC, USA) was dissolved in dimethyl sulfoxide (DMSO, Sigma-Aldrich, St. Louis, MO, USA) and stored at 4°C until used. ALI was induced by intranasal administration of LPS (Sigma-Aldrich, St. Louis, MO, USA) at 100 *μ*g in 20 *μ*L saline by drops for each mouse applied with a pipette as previously described [22, 23]. The control (vehicle) groups were injected i.p. with DMSO (100 *μ*L) after saline (20 *μ*L) treatment. The LPS groups were treated i.p. with sterile DMSO (100 *μ*L) following saline injection (20 *μ*L). The LPS + oxyberberine groups were treated i.p. with different sterile dosages of oxyberberine (i.p. 10, 20, and 50 mg/kg body weight) in DMSO (100 *μ*L) after saline injection (20 *μ*L). After the treatment, mice were killed by overdose of pentobarbital (i.p., 500 mg/kg sodium pentobarbital supplemented as needed) and deep anesthetization was confirmed by loss of the pedal withdrawal reflex.

### 2.3. Lung Pathology

The right lung samples were collected and fixed in 10% formaldehyde, paraffin embedded, and sliced into 4 *μ*m sections. Following H&E staining, pathological changes of the lung tissue samples were detected under a microscope. The pathological scores of lung tissues were evaluated according to lung injury, edema, and neutrophil infiltration as described previously [24]. The proinflammatory cytokines, including tumor necrosis factor *α* (TNF-*α*), interleukin 1*β* (IL-1*β*), and IL-6 were measured by ELISA kits according to the manufacturer's instruction (BioLegend, San Diego, CA, USA).

### 2.4. The Lung Wet/Dry Ratio

The right lung samples were collected and weighed to obtain the wet weight and then placed at 80°C for 48 h to obtain the dry weight. The wet/dry ratio was calculated as an indicator of pulmonary edema.

### 2.5. Myeloperoxidase Assay

Twenty-four hours after LPS administration, the lungs were excised and homogenized in myeloperoxidase (MPO) extractive phosphate buffer containing guaiacol and cetyltrimethylammonium bromide. After being subjected to centrifugation, the supernatant was reacted with hydrogen peroxide. The levels of MPO were indicated by absorbance at 470 nm [25].

### 2.6. BALF Analysis

BALF was harvested by washing the lung three times with 0.3 mL phosphate-buffered saline (PBS) (per time) through a tracheal cannula and then centrifuged at 3000 rpm for 10 min at 4°C. The cell-free supernatants were collected and divided into two portions. One portion was used to assess protein concentration by using a bicinchoninic acid (BCA) protein assay kit (Beyotime, Shanghai, China). Another portion was used to measure inflammatory cytokines as described above. In addition, the pellets were resuspended in 100 *μ*L PBS and were stained with Giemsa-Wright stain. Finally, the number of total cells and number of neutrophils were observed and recorded.

### 2.7. Western Blot Analysis

Western blot analysis was performed as described previously [26]. Briefly, proteins were separated by sodium dodecyl sulfate-polyacrylamide gel electrophoresis (SDS-PAGE) and transferred to polyvinylidene difluoride (PVDF) membranes. The membranes were incubated with primary antibodies against COX IV (11242-1-AP, ProteinTech, Wuhan, China), p62 (18420-1-AP, ProteinTech, Wuhan, China), Mfn2 (12186-1-AP, ProteinTech, Wuhan, China), and Parkin (ab77924, Abcam, Cambridge, MA, USA) at 4°C overnight. The membranes were incubated with secondary antibody for 1 h at room temperature. *β*-Actin was used as loading control. Immunoblots were visualized using enhanced chemiluminescence (ECL) (Thermo Scientific).

### 2.8. Immunofluorescence

The immunofluorescence was performed as previously described. Briefly, cells were treated with 4% formaldehyde for 30 min at room temperature and were permeabilized with 0.2% Triton X-100 (ABCone, Shanghai, China) for 2-5 min. After being blocked with 5% BSA for 30 min at room temperature, cells were then incubated overnight at 4°C with anti-Parkin primary antibody (ab77924, Abcam, Cambridge, MA, USA) and anti-TOMM20 primary antibody (11802-1-AP, ProteinTech, Wuhan, China). Then, cells were incubated with the secondary antibody. Immunofluorescence was observed under a fluorescence microscope (Olympus, Tokyo, Japan). Finally, Pearson's correlation coefficient was calculated to evaluate the colocalization of target proteins.

### 2.9. Flowcytometry

For cell apoptosis detection, cells were incubated in 5 *μ*L annexin V-FITC (Sigma-Aldrich, Munich, Germany) and 5 *μ*L propidium iodide (PI) (Sigma-Aldrich). For reactive oxygen species detection, cells were incubated in 10 *μ*M 2′-7′-dichlorodihydrofluorescein diacetate (DCFH-DA) (Sigma-Aldrich, Munich, Germany) [27]. After incubation, cells were examined on CytoFLEX flow cytometry (Beckman Coulter, USA).

### 2.10. Statistics

All data were expressed as mean ± SD, and all assays were performed at least in triplicate and experiments were repeated three times to verify the results for cell study. The statistics was carried out by using the GraphPad Prism software (version 5.0, USA). Comparison between groups was made using one-way analysis of variance followed by Tukey post test. *P* < 0.05 was considered statistically significant.

## 3. Results

### 3.1. Oxyberberine Alleviated Lung Injury Induced by LPS in Mice

Firstly, we evaluated whether oxyberberine has a protective effect on LPS-induced ALI. As shown in Figure 1(a), alveolar wall structures of lung tissues were intact from the control group mice. In contrast, a large amount of inflammatory cell infiltration and the alveolar wall thickened were shown in lung tissues from the LPS-treated group mice, which were significantly inhibited by oxyberberine pretreatment (Figure 1(a)). Notably, LPS induced a significant increase of the lung injury score. In the presence of oxyberberine, however, the LPS-induced increase of the lung injury score was significantly decreased (Figures 1(b) and 1(c)). These results suggest that oxyberberine could prevent the progress of ALI.

### 3.2. Oxyberberine Reduced Lung Edema, Neutrophils, and Inflammation in the Lung Tissues in LPS-Treated Mice

Next, we evaluated the effect of oxyberberine on the lung wet/dry ratio as an indicator of lung edema. As shown in Figure 2(a), the lung wet/dry ratio was significantly increased in the LPS-treated mice compared with the control mice. However, pretreatment with oxyberberine dose-dependently decreased the lung wet/dry ratio in LPS-treated mice.

Lung MPO activity was evaluated as an indicator of neutrophil accumulation in the lung.  Figure 2(b) shows that oxyberberine dose-dependently reduced MPO activation in the LPS-stimulated lung tissues.

We then evaluated the effect of oxyberberine on production of proinflammatory cytokines in lung tissue. As shown in Figures 2(c)–2(e), the levels of proinflammatory cytokines including TNF-*α*, IL-1*β*, and IL-6 were significantly increased when mice were treated with LPS. In contrast, oxyberberine dose-dependently inhibited the production of these proinflammatory cytokines in lung tissues from mice treated with LPS. These results suggest that oxyberberine prevented edema, neutrophils, and inflammation in LPS-treated mice.

### 3.3. Oxyberberine Reduced Edema, Neutrophils, and Inflammation in BALF in LPS-Treated Mice

Furthermore, we evaluated the changes of inflammation, edema, and neutrophils in BALF. Total protein was elevated in the BLAF from LPS-treated mice compared with control mice, and this increase was significantly reduced in mice treated with oxyberberine (Figure 3(a)).

The accumulation of inflammatory cells, such as neutrophils, was detected in the BALF. As shown in Figures 3(b) and 3(c), the number of total cells and number of neutrophils were significantly increased in the LPS-treated group mice compared with control mice. In contrast, oxyberberine treatment significantly inhibited the increased total cell number and neutrophils in BALF from mice treated with LPS.

Figures 3(d)–3(f) showed that oxyberberine dose-dependently inhibited the increased production of proinflammatory cytokines including TNF-*α*, IL-1*β*, and IL-6 in BALF from LPS-treated mice. These results further confirmed that oxyberberine prevented edema, neutrophils, and inflammation in LPS-treated mice.

### 3.4. Oxyberberine Inhibited LPS-Induced Mitophagy in A549 Cells

To explore the anti-inflammatory mechanism of oxyberberine, the potential effect of oxyberberine on mitophagy was assessed. As shown in Figures 4(a)–4(d), LPS significantly decreased the protein level of mitochondria proteins including COX IV, p62, and Mfn2. The translocation of Parkin was also assessed since it plays a critical role in mitophagy. Figures 4(e) and 4(f) shows that cytoplasmic Parkin was significantly decreased, whereas mitochondria significantly decreased in LPS-treated cells. As shown in Figure 5, LPS significantly increased the colocalization of TOMM20 and Parkin. In the presence of oxyberberine, however, the effect of LPS on the decreased expression of mitochondrial proteins, translocation of Parkin, and colocalization of TOMM20 and Parkin was significantly blocked. These results suggest that oxyberberine inhibited LPS-induced mitophagy in A549 cells.

### 3.5. Oxyberberine Inhibited LPS-Induced ROS, Inflammation, and Apoptosis in A549 Cells

Next, we evaluated the inhibitory effect of oxyberberine on LPS-induced apoptosis and ROS in A549 cells. As shown in Figure 6, flowcytometry assay shows that LPS significantly increased apoptosis and ROS production in A549 cells. Notably, the stimulatory effect of LPS was significantly inhibited by oxyberberine (Figure 6), suggesting that oxyberberine inhibited LPS-induced apoptosis and ROS production.

### 3.6. Inhibition of Mitophagy with Baf Prevented the Inhibitory Effect of Oxyberberine on LPS-Induced Mitophagy, Apoptosis, and ROS in A549 Cells

Then, we evaluated whether the inhibitory effect of oxyberberine involves mitophagy. Mitophagy was inhibited by lysosome inhibitor Baf. As shown in Figure 7, the inhibitory effect of oxyberberine on LPS-induced decrease of COX IV, p62, and Mfn2 was lost when mitophagy was inhibited by Baf. Meanwhile, in the presence of Baf, LPS failed to increase the colocalization of TOM20 and Parkin and oxyberberine showed no effect on the colocalization of TOM20 and Parkin (Figure 8). These results suggest that oxyberberine may inhibit LPS-induced mitophagy.

As expected, the inhibitory effect of oxyberberine LPS-induced apoptosis was almost totally lost when mitophagy was inhibited with Baf (Figures 9(a) and 9(b)). Similarly, the inhibitory effect of oxyberberine LPS-induced ROS production was lost in the presence of Baf (Figures 9(c) and 9(d)). These results suggest that oxyberberine inhibited LPS-induced apoptosis and ROS production through inhibition of mitophagy in A549 cells.

## 4. Discussion

In the present study, we investigated the potential protective effect of oxyberberine on ALI and the underlying mechanism.. Our results show that mitophagy was significantly increased in lung tissue of ALI mice, which was significantly inhibited by oxyberberine. In the presence of mitophagy inhibitor Baf, however, the inhibitory effect of oxyberberine was significantly attenuated. Our further *in vivo* study shows that oxyberberine inhibited lung pathological injury and prevented lung edema, as indicated by the changes of the lung wet/dry ratio and total protein levels in the BALF and inflammation in LPS-induced ALI mice. Therefore, the present study demonstrated that oxyberberine inhibited ALI through attenuation of mitophagy.

ALI is a life-threatening disorder with high morbidity and mortality worldwide. Although a great deal of effort has been put into the treatment of ALI, there is still lack of effective therapeutic strategy and no approved pharmacologic treatment for the regulation of the inflammatory response of this syndrome [28, 29]. LPS has been well accepted as the ideal model to explore the pathogenesis of ALI [30]. Lung edema derived from the disruption of the capillary-alveolar barrier is an important characteristic of ALI [31]. The lung wet/dry ratio is an indicator of pulmonary edema [29], and the total protein concentrations in the BLAF serve as a measurement of pulmonary vascular permeability [32]. Our results demonstrated that LPS stimulation led to an increased lung wet/dry ratio and elevated inflammatory cell count in the BALF. These results suggest that ALI was successfully established.

The commonly prescribed therapeutics for inflammatory diseases includes corticosteroids, immunosuppressive agents, and nonsteroidal anti-inflammatory drugs (NSAIDs). Berberine (BBR), a quaternary isoquinoline alkaloid derived from traditional Chinese medicinal herbs like *Coptidis chinensis* Franch., is commonly used as a nonprescription drug to treat gastroenteritis, colitis, diarrhea, and dysentery [8]. In the liver, berberine is metabolized by oxidative demethylation and glucuronidation to berberrubine, thalifendine, demethyleneberberine, jatrorrhizine, and their corresponding glucuronides [33]. Of note, oxyberberine is a nature oxoderivative of berberine, which exerted strong anti-inflammatory effects. staff-cmt="Please consider rephrasing the highlighted part for clarity purposes." author-reply="Please replace the highlighted part with "For example, Li et al. reported that the anti-inflammatory effect of Rhizoma Coptidis was mainly from oxyberberine. [12]. Furthermore, they further demonstrated that the intestinal microflora could transform berberine into oxyberberine by oxidation reaction and play a protective role in ulcerative colitis [8]. In consistency with these findings, the present study demonstrated that oxyberberine prevented apoptosis and inflammation in LPS-induced ALI.

There are accumulating data showing that mitophagy was increased in acute heart damage [34], acute kidney damage [35], and acute lung injury [36]. Mitophagy can have beneficial effects during acute organ damage. However, excessive mitophagy may promote mitochondrial dysfunction and cause cell injury and death [37]. For example, it has been reported that mitophagy contributes to increased inflammation and lung injury in ALI [36, 38]. During ALI, the activation of mitophagy plays a critical role in the production of proinflammatory cytokines including TNF-*α*, IL-1*β*, and IL-6 and these cytokines all play important roles in the progress of ALI [39, 40]. Another study by Luo et al. reported that mitochondrial division inhibitor 1 (Mdivi-1) attenuates mitophagy and mitigates LPS-induced apoptosis, oxidative stress, and inflammation in ALI [38]. In consistency with these findings, the present study shows that mitophagy was increased in ALI and that oxyberberine significantly inhibited LPS-induced ALI. Considering the potent protective effect of oxyberberine, the present study may provide solid basis for its clinical usage.

The Parkin-Pink1 signaling pathway plays an important role in mitophagy. For example, it has been reported that Parkin-Pink1-mediated mitophagy contributes to necroptosis and pathology in chronic obstructive pulmonary disease (COPD) [37]. During ALI, Parkin/Pink1-mediated mitophagy contributes to inflammation [36]. In consistency with these studies, we discovered that oxyberberine prevented LPS-induced ALI through inhibition of mitophagy. In contrast, another study demonstrated that Parkin-Pink1-mediated mitophagy alleviated the stimulator of interferon gene- (STING-) induced inflammation [41]. These studies demonstrated that Parkin-Pink1-mediated mitophagy may have a detrimental or protective role in different stimulations and in different cells.

In summary, the present study demonstrated that oxyberberine inhibited the inflammatory response through inhibition of Parkin/Pink1-mediated mitophagy in LPS-induced ALI. This finding suggests that oxyberberine may have pharmacological application in the prevention and treatment of ALI.

## Figures and Tables

**Figure 1:** Oxyberberine inhibited LPS-induced acute injury. Representative H&E images (a) and summarized lung injury scores (b) showing the dose-dependent protective effect of oxyberberine on LPS-induced ALI. Data were expressed as mean ± SD (*n* = 5–6). ^∗∗^*P* < 0.01 and ^∗∗∗^*P* < 0.001 vs. the control group; ^##^*P* < 0.01 vs. the LPS group.

**Figure 2:** Oxyberberine inhibited edema, neutrophils, and inflammation in lung tissue of LPS-treated mice. Summarized data showing the inhibitory effect of oxyberberine on the increased wet/dry ratio (a) and MPO activity (b) in LPS-induced ALI. Summarized data showing the inhibitory effect of oxyberberine on the increased production of proinflammatory cytokines including TNF-*α* (c), IL-1*β* (d), and IL-6 (e) in LPS-induced ALI. Data were expressed as mean ± SD (*n* = 5–6). ^∗^*P* < 0.05, ^∗∗^*P* < 0.01, and ^∗∗∗^*P* < 0.001 vs. the control group; ^##^*P* < 0.01 vs. the LPS group.

**Figure 3:** Oxyberberine reduced edema, neutrophils, and inflammation in BALF in LPS-treated mice. Summarized data showing the inhibitory effect of oxyberberine on the increased total protein (a), cell count (b), neutrophils (c), TNF-*α* (d), IL-1*β* (e), and IL-6 (f) in BALF in LPS-induced ALI. Data were expressed as mean ± SD (*n* = 5–6). ^∗^*P* < 0.05, ^∗∗^*P* < 0.01, and ^∗∗∗^*P* < 0.001 vs. the control group; ^##^*P* < 0.01 and ^###^*P* < 0.001 vs. the LPS group.

**Figure 4:** Oxyberberine inhibited LPS-induced mitophagy in Western blot assay in A549 cells. Representative Western blot images (a) and summarized data (b, c, d) showing the inhibitory effect of oxyberberine on the changes of COX IV, P62, and Mfn2 in A549 cells with or without LPS and oxyberberine treatment. RepresentativeWestern blot images and summarized data showing the Parkin protein level in cytoplasm (e) and mitochondria (f) in A549 cells with or without LPS and oxyberberine treatment. Data were expressed as mean ± SD (*n* = 4–6). ^∗^*P* < 0.05 and ^∗∗^*P* < 0.01 vs. the control group; ^#^*P* < 0.05 vs. the LPS group.

**Figure 5:** Oxyberberine inhibited LPS-induced mitophagy in immunofluorescence assay in A549 cells. Representative immunofluorescence images (a) and summarized data showing the inhibitory effect of oxyberberine on the colocalization of TOMM20 and Parkin in A549 cells with or without LPS treatment. Data were expressed as mean ± SD (*n* = 5–6). ^∗∗^*P* < 0.01 vs. the control group; ^##^*P* < 0.01 vs. the LPS group.

**Figure 6:** Oxyberberine inhibited LPS-induced apoptosis and ROS production in A549 cells. Representative flowcytometric images (a) and summarized data (b) showing the inhibitory effect of oxyberberine on LPS-induced apoptosis. Representative flowcytometric images (c) and summarized data (d) showing the inhibitory effect of oxyberberine on LPS-induced superoxide production. Data were expressed as mean ± SD (*n* = 5–6). ^∗∗∗^*P* < 0.001 vs. the control group; ^###^*P* < 0.001 vs. the LPS group.

**Figure 7:** Inhibition of mitophagy with Baf prevented the inhibitory effect of oxyberberine on LPS-induced mitophagy in Western blot assay in A549 cells. Representative Western blot images (a) and summarized data showing that Baf prevented the inhibitory effect of oxyberberine on LPS-induced decrease of COX IV (b), P62 (c), and Mfn2 (d). Representative Western blot images and summarized data showing the Parkin protein level in cytoplasm (e) and mitochondria (f) in A549 cells with or without LPS, Baf and oxyberberine treatment. Data were expressed as mean ± SD (*n* = 4–6). ^∗^*P* < 0.05 vs. the control group.

**Figure 8:** Baf prevented the inhibitory effect of oxyberberine on LPS-induced colocalization of TOMM20 and Parkin in A549 cells. Representative immunofluorescence images (a) and summarized data (b) showing that Baf prevented the inhibitory effect of oxyberberine on LPS-induced colocalization of TOMM20 and Parkin. Data were expressed as mean ± SD (*n* = 5–6).

**Figure 9:** Inhibition of mitophagy with Baf prevented the inhibitory effect of oxyberberine on LPS-induced apoptosis and ROS production in A549 cells. Representative flowcytometric images (a) and summarized data (b) showing that Baf prevented the inhibitory effect of oxyberberine on LPS-induced apoptosis. Representative flowcytometric images (c) and summarized data (d) showing that Baf prevented the inhibitory effect of oxyberberine on LPS-induced superoxide production. Data were expressed as mean ± SD (*n* = 5–6). ^∗∗∗^*P* < 0.001 vs. the control group.

## Data Availability

The datasets used and analyzed during the current study are available from the corresponding author on reasonable request.
